# Evaluation of Liquid Biopsy in Patients with HER2-Positive Breast Cancer

This article has been retracted.

**DOI:** 10.1155/2021/6388492

**Published:** 2021-12-03

**Authors:** Jianguo Huai, Ming Cao, Yan Jiang, Xiaomiao Yang, Yanyan Zhu, Youyi Si, Man Xu, Chenxiang Shen, Tao Han, Xiaochun Lian

**Affiliations:** ^1^Department of Pathology, Wuhu No. 1 People's Hospital, Wuhu 241000, China; ^2^Department of Breast Surgery, Wuhu No. 1 People's Hospital, Wuhu 241000, China

## Abstract

Breast cancer is one of the common malignant tumors, and liquid biopsy has become a hot spot for clinical testing. To clarify the detection effect of liquid biopsy in breast cancer, we collected peripheral blood of HER2-positive (human epidermal growth factor receptor 2-positive) patients. Circulating tumor cells (CTCs) were isolated and analyzed. HER2 expression on CTCs was detected. The results showed that in the 198 HER2-positive samples, the CTC detection rate was 79.8% (158/198), and the mean number of CTCs was 21, ranging from 1 to 63/7.5 mL peripheral blood. Only 41.1% (65/158) of patients had histology and CTC HER2 status consistent with the remaining 58.9% (93/158) of patients, although their histological HER2 was positive, and CTC HER2 was negative. Our study confirmed the value of CTC HER2 real-time status testing in HER2-positive breast cancer patients. The inconsistency in HER2 status between CTCs and histology may be related to the time interval between CTCs and histological HER2 detection, suggesting that real-time HER2 detection is necessary for histological HER2-positive patients.

## 1. Introduction

Breast cancer is one of the most common female tumors, and GLOBOCAN predicts that there will be 210,000 new cases of breast cancer in China in 2020 [1]. The occurrence and development of breast cancer is regulated by multiple genes. In many markers related to breast cancer, estrogen receptor (ER), progesterone receptor (PR), human epidermal growth factor receptor 2 (HER2), and Ki-67 are considered to be the markers for breast cancer [2, 3]. The expressions of ER, PR, HER2, and Ki-67 directly determine the choice of treatment. HER2 is a very important molecular marker for breast cancer. About 20% of newly diagnosed breast cancer patients are HER2-positive [4, 5]. The main difficulty in tumor treatment is that the cause is complex and constantly changing, and the etiology is complex and constantly changing, and the status of the drug target is not 100% predictive of efficacy [6, 7]. Therefore, for more accurate and effective treatment, it is necessary to evaluate the efficacy in a timely manner and adjust the treatment strategy in a timely manner. However, traditional evaluation methods do not meet the above requirements [8–10].

Currently, the HER2 status of breast cancer patients is mainly determined by immunohistochemical (IHC) detection and fluorescent in situ hybridization (FISH) on a section of tumor tissue obtained by surgery or needle biopsy. In this context, liquid biopsy has become a hot spot for clinical testing. Liquid biopsy is a diagnostic analysis through body fluid samples. The types of body fluids that have been reported for liquid biopsy include peripheral blood, pleural and ascites fluid and cerebrospinal fluid in disease states, urine, and saliva [11]. CTCs, which can be used for liquid biopsy in peripheral blood, have been widely used in clinics as a biomarker of liquid biopsy, and it is an important marker in the process of tumor metastasis. Moreover, CTCs have been confirmed to be widely present in the peripheral blood of people suffering from breast cancer [12]. The main advantage of liquid biopsy is that it is small in trauma and very convenient for real-time dynamic monitoring. In addition, in the liquid state, the components of various tumor sources are relatively uniform, which can reflect the heterogeneity of the tumor in time and space from a holistic perspective.

In this study, we mainly conducted research on CTCs, collected the peripheral blood of HER2-positive patients, separated and analyzed CTCs, and detected HER2 expression on CTCs, then selected CTCs HER2-positive patients to test the expression of ER, PR, and Ki-67 in order to have a clearer concept of liquid biopsy for its better application in clinic in the future and better guide individualized treatment of such patients.

## 2. Materials and Methods

### 2.1. Specimen Source

There are collected breast cancer samples from March 2017 to March 2019 in Wuhu First People's Hospital. Histologically, HER2-positive patients who are defined by the IHC or FISH were enrolled in the present study. The criteria for inclusion were female patients; tumor diameter ≥ 2 cm; no chemotherapy, endocrine therapy, radiotherapy, and targeted therapy [13]. Patients sign a written informed consent form. According to the inclusion criteria, 198 patients with breast cancer were enrolled, aged 29-84 years. We then analyzed 7.5 mL of these samples for CTC content using a Cyttel® (Jiangsu, China) immunofluorescence in situ hybridization (imFISH) approach.

### 2.2. CTCs Collection and Processing

7.5 mL peripheral blood was added to the centrifuge tube, 6.5 mL of buffer was added, and the mixture was mixed and centrifuged at 800 g for 10 min. The sample was placed in the AutoPrep system, and the parameters were set according to the instruction manual. After the treatment, the sample was transferred to the MagNest device, incubated for 20 min or more in the dark, and the MagNest was placed in the AnalyZer for fluorescence scanning [14]. The CTC positive standard is CK positive and conforms to cell morphology, DAPI (Sigma-Aldrich, USA) is positive, and the signal is in the range of CK. HER2 expression on CTCs was assessed by staining the cells with a FITC-labeled anti-HER2 antibody (Veridex LLC, USA). For the time when CTCs were positive, its expression was defined as 0 (no expression), 1+ (weak expression), 2+ (moderate expression), and 3+ (strong expression) according to the fluorescence intensity of HER2. Those patients with >30% of CTCs overexpressing HER2 (3+) were defined as CTC HER2-positive [15].

### 2.3. Immunohistochemical Testing

The antibody used was produced by Maixin Co., and the sample was applied to the machine after 1 hour of baking. It was automatically stained with Roche Immunohistochemistry (Roche Diagnostics, Germany). After the procedure was completed, it was washed, dehydrated, and transparently sealed with xylene.

### 2.4. Immunofluorescence

Frozen tumor tissue slices of 5 mm thickness were fixed with cold acetone for 10 min, washed with PBS, and then, blocked with 10% donkey serum for 45 min at room temperature. Slices were then incubated overnight with pertuzumab (ThermoFisher Scientific, USA) at 4°C [16]. Next, sections were further stained with AlexaFluor488-labeled goat anti-human antibody (ThermoFisher Scientific, USA). A coverglass was applied to each slide using Vectashield mounting medium (Vector Laboratories, Burlingame, CA, USA), and imaging was performed using an A1R confocal microscope (Nikon, Nikon Instruments, Melville, NY, USA).

### 2.5. FISH Test

The sample was dewaxed by xylene, dehydrated by 100%, 85%, and 70% alcohol gradient, and then, treated with pretreatment solution for 20 minutes. After digestion with a protease solution, it was naturally air-dried and incubated with a probe. The mixture was heated at 85°C for 5 min in a Thermo Brite hybridization (Abbott Molecular, USA) apparatus and reacted overnight at 37°C. The next day, the unbound probe was washed with a constant temperature buffer, dehydrated by alcohol gradient soaking, air-dried, and DAPI counterstain solution was titrated on a glass slide and sealed.

### 2.6. Statistical Analysis

Fisher's exact test was used to analyze whether there were differences in clinical features between patients with CTC = 0 and CTC 1 and between patients with CTC HER2-positive and CTC HER2-negative based on histology and time of CTC HER2 testing. Patients were divided into different groups by interval, and differences in HER2 state consistency among different groups were analyzed by chi-square test. *P* values < 0.05 was considered statistically significant, and SPSS 23.0 (IBM Corporation, USA) was used for all analyses.

## 3. Results

### 3.1. Patient Characteristics and CTC Detection

From March 2017 to March 2019, a total of 198 HER2-positive breast cancer patients were enrolled, with an average age of 49 years (29-84 years). The results of immunohistochemistry and immunofluorescence showed that the HER2 protein was mainly expressed in the cell membrane of breast cancer, which was brown (Figures 1(a) and 1(b)). According to patient's CTC test value, the patients were divided into CTCs ≥ 1 group and CTCs = 0 group. The clinical characteristics of these two groups of patients are shown in Table 1. The overall CTC detection rate was 79.8% (158/198), and the mean number of CTCs was 21, ranging from 1 to 63/7.5 mL peripheral blood. The frequency distribution histogram of CTCs is shown in Figure 2. The lymph node and pathological stage between the CTC detection group and the undetected group were statistically significant (*P* < 0.05).

### 3.2. HER2 Status on CTCs

The HER2 expression on each CTCs is defined as 0, 1+, 2+, or 3+. 0 is no signal, 1+ is a faint signal, 2+ is ambiguous, and 3+ is a clear and clear signal. Using our CTC HER2 positive criteria, >30% of CTCs were strongly expressed by HER2 (3+), and only 41.1% (65/158) of patients had consistent histology and CTC HER2 status, with the remaining 58.9% (93/158) patients, although their histology HER2 was positive, and CTC HER2 was actually negative (Table 2). In the ER and/or PR positive group, the HER2 inconsistency rate between tissue and CTCs was 74.7% (118/158).

### 3.3. Expression of ER, PR, and Ki-67 on CTCs

The analysis included a total of 158 CTC-positive patients, estrogen receptor (ER) positive in 98 (62.0%) patients, and progesterone receptor (PR) positive in 75 (47.5%) patients. In 88 (55.7%) patients, the Ki-67 positive rate was greater than 50% (Figure 3). The expression of ER, PR, and Ki-67 can be well detected on CTCs as a real-time dynamic detection, providing guidance for subsequent personalized medication and cancer surveillance.

## 4. Discussion

There is increasing evidence that HER2 status in breast cancer patients changes during treatment. CTCs can provide a HER2 real-time detection solution with minimally invasive and simple advantages [17, 18]. Although this application is very promising, there are many CTC detection methods and different CTCS HER2-positive standards, which greatly affect the use of CTC HER2 detection in clinical practice to guide HER2-targeted therapy. Histologically, HER2-positive conversion to CTCs-HER2 negative seems to be a very common phenomenon [19, 20]. In this study, this data was 58.9% (93/198), and the results of previous studies were 41.7% (5/12), 45.5% (5/11), and 50% (1/2) [21–23]; the results of this study are similar to those of other literatures. This high degree of inconsistency further underscores the need and urgency of real-time HER2 detection. Especially in developing countries like China, high medical expenses have always been a huge burden for patients. By CTC testing, patients with histological HER2-positive but CTC HER2-negative patients can avoid overtreatment of HER2-targeted drugs and save costs. One problem with this study was that all CTC data were based on a single-sample test, and no CTC analysis was performed during follow-up of patients. In future studies, CTC analysis during follow-up is necessary because the number of CTCs and the status of HER2 will also change over time.

At present, the detection in breast cancer patients is mainly immunohistochemical technology. The detection of ER, PR, Ki-67, and other expression in breast cancer is very important [24]. The detection of these indicators can not only make the diagnosis of lesions but also choose the basis for personalized treatment. The ER protein is present in the cells of the target organ and can specifically bind to the hormone to form a hormone-receptor complex, so that the hormone exerts its biological effects. ER can bind to its ligand to regulate the proliferation, survival, and invasion of tumor cells and the formation of tumor angiogenesis. PR is a member of the steroid hormone receptor family. Ki-67 is an effective indicator of cell proliferation [6, 25–27]. These three indicators serve as indicators of proliferation and activity of breast cancer cells and are used for the selection of subsequent treatment options. In this study, a total of 158 CTC-positive patients were positive for estrogen receptor (ER) in 98 (62.0%) patients and progesterone receptor (PR) positive in 75 (47.5%) patients. The Ki-67 positive rate was greater than 50% in 88 (55.7%) patients. The results of this experiment show that CTCs can be used as real-time dynamic detection to provide guidance for subsequent personalized medication and cancer surveillance.

## 5. Conclusion

In summary, our study demonstrated the value of CTC HER2 real-time status detection in HER2-positive breast cancer patients. The inconsistency of HER2 status between CTCs and histology may be related to the time interval between the detection of CTCs and histological HER2, suggesting that real-time detection of HER2 is very necessary for patients with positive histological HER2.

## Figures and Tables

**Figure 1:** Expression of HER2 protein in breast cancer tissues. (a) Immunohistochemistry and (b) immunofluorescence used to display the HER2 protein expression in breast cancer tissues.

**Figure 2:** Frequency distribution histogram of CTCs.

**Figure 3:** Status of ER, PR, and Ki67 in CTC-positive patient.

**Table 1:** Clinical characteristics of all patients.

Characteristics	Total	CTC = 0 (%)	CTC ≥ 1 (%)	*P*
Total *n* (100%)	198	40 (20.2%)	158 (79.8%)	
Age (years)				
Median	49	49	49	0.546
Range	29-84	29-84	30-79	
ER and/or PR				
Positive	158	32 (20.3%)	126 (79.7%)	0.012
Negative	40	8 (20.0%)	32 (80.0%)	
TNM stage				
II	71	28 (39.4%)	43 (60.6%)	0.036
III	127	12 (9.4%)	115 (90.6%)	
No. of metastasis				
1	38	22 (57.9%)	16 (42.1%)	0.085
≥2	160	18 (11.3%)	142 (88.7%)	
Number of CTCs			21 (1-63/7.5 mL)	

**Table 2:** Comparison of CTCs, primary tumor by HER2 status in patients.

	Total	CTCs-HER2-positive *n* (%)	CTCs-HER2-negative *n* (%)
Primary-HER2 status	198	158 (79.8%)	40 (20.2%)
Positive	158	65 (41.1%)	93 (58.9%)
Negative	40	18 (45.0%)	22 (55.0%)

## Data Availability

The data used to support the findings of this study are included within the article.
